# Nodal Enhances Perineural Invasion in Pancreatic Cancer by Promoting Tumor-Nerve Convergence

**DOI:** 10.1155/2022/9658890

**Published:** 2022-01-27

**Authors:** Sugang Shen, Qiqi Wang, Xueni Wang, Jiachun Ding, Fan Chen, Ying Xiao, Tao Qin, Weikun Qian, Jiahui Li, Qingyong Ma, Jiguang Ma

**Affiliations:** ^1^Department of Hepatobiliary Surgery, The First Affiliated Hospital of Xi'an Jiaotong University, Xi'an 710061, China; ^2^Department of General Surgery, The Second Hospital of Shanxi Medical University, Taiyuan 030001, China

## Abstract

Perineural invasion (PNI) is a typical feature of pancreatic ductal adenocarcinoma (PDAC), which occurs in most cases. The embryonic protein Nodal plays a critical role in embryonic neural development and is overexpressed in human pancreatic cancer. In this study, we explored the contribution of Nodal to pancreatic cancer PNI and progression. We evaluated the function of Nodal in PNI by coculturing rat dorsal root ganglia and pancreatic cancer cells in vitro and performing cellular and molecular biology assays. The results illustrate that Nodal upregulates NGF (nerve growth factor), BDNF (brain-derived neurotrophic factor), and GDNF (glial cell line-derived neurotrophic factor) expression in pancreatic cancer cells and promotes cancer cell migration/invasion. Furthermore, in the in vitro 3D PNI model, Nodal enhances nerve outgrowth to pancreatic cancer cell colonies. Our study indicates that Nodal participates in tumor invasion by mediating neural and tumor cell signaling interactions, and inhibiting the expression of Nodal represents a potential strategy for targeting PNI in pancreatic cancer therapy.

## 1. Introduction

Pancreatic cancer (PC) is one of the most lethal cancers with a dismal 5-year survival rate of about 10% [1]. In particular, pancreatic ductal adenocarcinoma (PDAC) is the most common histological type with highly invasive and metastatic properties. Its poor prognosis is due to late diagnosis, early metastasis, and limited treatment options, which result in roughly equal mortality and morbidity in PC patients [2, 3]. Although surgical resection is considered the only possible cure for PC, only 20% of pancreatic cancer patients can undergo curative resection [4]. Postoperative recurrence is the main factor leading to surgical failure, which occurs in up to 60% of patients. With current multimodal treatment, the median overall survival is only 11 months [5, 6].

Recent studies have found that perineural invasion (PNI) is a common feature of PC with an incidence of 87% [7–9]. PNI is characterized by tumor cell invasion in, around, and through the nerves while encroaching on at least 33% of its circumference or within any of the 3 layers of the nerve sheath [10]. PNI is an independent risk factor for disease-free survival (DFS) and/or OS and can be used as a prognostic indicator. The absence of PNI has an independent protective effect on the long-term survival (more than 10 years) of PDAC patients. Whether pancreatic cancer patients are accompanied by PNI is one of the key references for guiding personalized antitumor treatment plans [9]. PNI has been found in the early stages of pancreatic cancer and is related to pain [11, 12], local recurrence [13], metastasis [14, 15], and poor prognosis [14]. Despite extensive knowledge of the clinical significance of PNI, its pathogenic mechanism remains unknown.

Nodal is a type of embryonic morphogen and a member of the transforming growth factor (TGF) beta superfamily. In humans, the Nodal gene is located on chromosome 10 and contains three protein-coding exon regions that are translated into a 347-amino acid proprotein. Nodal plays a crucial role during early embryonic development and is almost undetectable in normal human cells. During embryogenesis, Nodal signaling activates the differentiation process and eventually loses function after transcriptional silence [16]. Nodal signaling plays an important role during neural development. Nodal influences neural tube closure by adjusting N-cadherin levels in zebrafish [17]. Deficiencies in the Nodal signaling pathway potentially underlie human neural tube defects, such as exencephaly, a fatal condition characterized by an open neural tube in the anterior brain. Furthermore, numerous studies have revealed Nodal re-expression in several tumor types. The acquisition of Nodal expression is directly related to tumorigenesis, proliferation, invasion, and metastasis, EMT (epithelial-mesenchymal transition), and angiogenesis [16, 18].

Previous studies of Nodal in pancreatic cancer focused on its role in promoting stem cell-like phenotypes [18]. However, the effect of Nodal on pancreatic cancer PNI remains unclear. In this study, we hypothesized that high expression of Nodal promotes nerve infiltration and local invasion of pancreatic cancer. The expression of neurotrophins is enhanced by Nodal and then promotes the growth of synapses toward pancreatic cancer cells. Besides, Nodal promotes the production of matrix metalloproteinases (MMPs), thereby promoting PNI via reducing the resistance of interstitial spaces between tumor cells and nerves.

## 2. Materials and Methods

### 2.1. Cell Lines, Culture Conditions, and Reagents

The human PC cell lines (BxPC3 and Panc-1) were obtained from the Chinese Academy of Sciences Cell Bank of Type Culture Collection, and they were cultured in the corresponding medium (Invitrogen) which contains 10% fetal bovine serum (FBS), 100 *μ*g/ml penicillin-streptomycin. The cells were incubated at 37°C in a humidified atmosphere containing 5% CO_2_. Antibodies were purchased from the following sources: recombinant mature human Nodal (rhNodal) (R&D Systems) and its inhibitor SB431542 (Sigma-Aldrich); anti-MMP-9 (Bioworld); and anti-NGF, anti-BDNF, and anti-GDNF (Abcam).

### 2.2. Immunofluorescence

Panc-1 and BxPc-3 were fixed in 4% paraformaldehyde for 20 min, and 3% H_2_O_2_ was added to quench the activity of endogenous peroxidase. Then, the samples were permeabilized with 0.5% Triton *X* 100 for 5 min and blocked with bovine serum albumin for 15 min at room temperature. Next, PC cells were incubated with the primary antibody at 4°C (overnight) and fluorescein-conjugated secondary antibodies (Jackson) for 1 h. DAPI was used to stain the nuclei for 5 min. The images were collected by a fluorescence microscope (Nikon).

### 2.3. RNAi Transfections

siRNA against Nodal (5′-AGACAUGAUCGUGGAAGAAtt-3′) and negative control (5′-CAUUUCGUCUGCCUCAUAUtt-3′) were purchased from GenePharm. Transfection was performed with Lipofectamine RNAi MAX Reagent (Invitrogen) according to the manufacturer's instructions. After 48 h of transfection, the cells were used for further experiments.

### 2.4. Enzyme-Linked Immunosorbent Assay (ELISA)

Cells were treated with corresponding agents for 24 h and then cultured in an FBS-free medium for 72 h. Then, the culture medium was collected and centrifuged at 1500 rpm for 5 min to remove particles. The supernatant was frozen at −80°C. The production of NGF in the supernatant was detected using a commercial ELISA kit (R&D Systems) according to the manufacturer's instructions.

### 2.5. Western Blotting Analysis

Cells were lysed using RIPA which contained protease inhibitors (Roche). Relative proteins were resolved on a denaturing SDS polyacrylamide gel by electrophoresis and electrotransferred onto nitrocellulose membranes. The membranes were blocked with 5% nonfat dry milk for 2 h. Then, the membranes were incubated with corresponding primary antibodies against NGF, BDNF, GDNF, MMP-9, and *β*-actin (4°C, overnight) and hybridized to the appropriate secondary antibodies (room temperature, 1 h). *β*-actin served as the loading control. The probed proteins were detected by enhanced chemiluminescence (Millipore).

### 2.6. Cell Invasion Assay

The Transwell chamber (8.0 *μ*m; Millipore) which was coated with 30 *μ*l of Matrigel was placed into a 24-well culture plate. 5×10^4^ PC cells were resuspended in DMEM (containing 1% FBS) with or without rhNodal and seeded in the upper chamber. Furthermore, 600 *μ*l of DMEM medium (containing 20% FBS) was added to the lower chamber. The Transwell chamber was incubated for 24 h. Cells were fixed in methanol and stained with crystal violet. The number of invasion cells was counted under a light microscope (Nikon) in 10 randomly selected fields.

### 2.7. Dorsal Root Ganglion (DRG) Coculture Assay

Newborn rats were purchased from the Animal Center of the Medical College of Xi'an Jiaotong University and were sacrificed using carbon dioxide and sterilized with 75% ethanol. DRGs from the lumbar areas were dissected, stripped of meninges and nerve stumps, and then implanted into a drop of 50% Matrigel (BD Biosciences). After solidification, DMEM/F12 (containing 10% FBS) with or without rhNodal and/or Nodal inhibitor (SB431542) was carefully added, which was changed every 3 days under routine culture. Images were photographed by a light microscope (Nikon). For evaluating the coculture model, we defined the minimum distance between the edge of the cancer cells and the edge of DRG as parameter *γ*, the migration distance of cancer cells toward DRG as parameter *α*, and the DRG outgrowth length toward cancer cells as parameter *β*. Here, the invasion index = *α*/*γ*, and the DRG outgrowth index = *ß*/*γ* (Figure 1(d)). The migration distance was measured by the abovementioned images.

### 2.8. Statistical Analyses

For statistical analyses, the SPSS 13.0 software package was adopted. All the data were described by mean ± standard deviation (SD). The differences between the enumeration data were determined using the Pearson correlation coefficient or Fisher's exact test. The differences between measurement data were determined using analysis of variance (ANOVA) followed by Bonferroni's correction for multiple comparisons. *P* < 0.05 was considered significant.

## 3. Results

### 3.1. Nodal Increases the Expression of Neurotrophins and Enhances Pancreatic Cancer Cell Invasion

To determine whether Nodal affects the expression of neurotrophins (NGF, BDNF, and GDNF) and MMP-9 in pancreatic cancer cells, Panc-1 and BxPC-3 cells were treated with rhNodal (0, 50, and 100 *μ*M) for 24 h. Western blot analysis was used to evaluate NGF, BDNF, GDNF, and MMP-9 protein expression in pancreatic cancer cells. The results revealed that rhNodal increased the expression levels of NGF, BDNF, GDNF, and MMP-9 in a dose-dependent manner (Figure 2(a)). Furthermore, immunofluorescence results showed that NGF levels were markedly increased in Panc-1 and BxPC-3 cells following treatment with rhNodal (100 *μ*M) for 24 h (Figure 2(b)). ELISA results confirmed that NGF secretion increased in Panc-1 cells treated with rhNodal (0, 50, and 100 *μ*M), which is consistent with western blot results (Figure 2(c)). To elucidate the role of Nodal in pancreatic cancer cell invasion, Transwell chamber assays with Matrigel were performed. In the Transwell invasion assays, the invasion ability of pancreatic cancer cells treated with rhNodal (100 *μ*M) was enhanced compared with the control group (Figure 2(d)). These data suggested that high Nodal expression levels upregulated neurotrophins and MMP-9 expression levels and subsequently increased pancreatic cancer cell invasion.

### 3.2. Nodal Knockdown Decreases the Expression of Neurotrophins and Inhibits Pancreatic Cancer Cell Invasion

To determine whether Nodal influences the expression of neurotrophins and invasion ability, we used Nodal siRNA to knock down Nodal. Three siRNA sequences were designed, and the efficiency of these siRNAs was evaluated by western blot (Figure 3(a)). SiRNA2 was selected for further experiments given its high-quality effect on knockdown the expression of Nodal. We found that the expression of neurotrophins (NGF, BDNF, and GDNF) and MMP-9 in Panc-1 and BxPC-3 cells was significantly decreased in the siNodal group compared to the siNC group (Figure 3(b)). Immunofluorescence results showed that NGF expression was reduced in pancreatic cancer cells after Nodal knockdown, and these results were consistent with western blot results (Figure 3(c)). In the Transwell invasion assays, siNodal inhibited the invasion ability of Panc-1 and BxPC-3 cells (Figure 3(d)). These data further proved that Nodal expression levels can influence neurotrophins and MMP-9 expression.

### 3.3. Nodal Inhibition Hampers the Infiltrative Growth of DRG Synapses

To investigate whether Nodal affects DRGs' growth, DRGs were extracted from newborn rats and cultured in 24-well plates. Nodal with or without its inhibitors was added into the culture solution which was changed every two days to maintain the drug concentration in the culture solution. The outward growth of ganglion synapses was observed and recorded under a microscope every day. After 96 h of culture, the outward growth of DRG synapses in the rhNodal group was enhanced compared with that in the control group, but no significant difference was noted. However, upon inhibition of Nodal by SB431542, the outward growth of DRGs was significantly reduced compared with the rhNodal group (Figure 4). These data indicate that Nodal is a necessary but insufficient condition to cause synaptic growth.

### 3.4. Nodal Affects the Interaction between Pancreatic Cancer Cells and DRGs

We further wanted to demonstrate whether Nodal accelerates PNI of pancreatic cancer cells. An in vitro peripheral neural invasion model was created using pancreatic cancer cells with DRGs in Matrigel according to previous reported models [19, 20]. During the coculture period of pancreatic cancer cells (Panc-1 and BxPC-3) and DRGs, we found that the DRG synaptic boundary and pancreatic cancer cell boundary moved toward each other more obviously in the Nodal intervention group than in the control group. After 96 hours of coculture, the DRG outgrowth ratio and tumor invasion index were calculated. The calculation method of DRG growth rate and tumor invasion index refers to a previously reported method (Figure 1(d)) [21]. The DRG outgrowth ratio and tumor invasion index of the rhNodal group increased faster than the control group (Figures 1(a) and 1(c)). The trend of growth between DRGs and pancreatic cancer cells was inhibited when Nodal was knockdown in pancreatic cancer cells by small interfering RNA (Figure 1(b)). Besides, the DRG outgrowth ratio and tumor invasion index were reduced in the siNodal group compared to those in the NC group (Figure 1(c)). The abovementioned results prove that Nodal acts on tumor cells, thereby affecting the interaction between tumor cells and DRGs.

## 4. Discussion

Members of the TGF*β* family, including bone morphogenetic proteins (BMPs), TGF*β*, and Nodal/activin, whose functions vary with the cellular environment (including disease, local environment, and the characteristics and dosage of the ligand). As a versatile cytokine, TGF*β* is proved to promote invasion and metastasis in many tumors. Our previous studies have shown that, as an activator of mesenchymal cells, TGF*β* affects YAP expression, which in turn mediates CTGF (connective tissue growth factor) expression and activation of pancreatic cancer stellate cells [22]. In the tumor microenvironment, Schwann cells are an important source of TGF*β* in PDAC, and TGF*β* signal activation in PDAC samples is positively correlated with peripheral infiltration [23]. Nodal and activin bind to their coreceptors, activin-like (Alk) type I receptors Alk4/7, and Cripto-1 constitutes an important coreceptor for Nodal signaling. Recent studies showed that Nodal is aberrantly upregulated in many cancers, such as prostate cancer, bladder cancer, breast cancer, and colon cancer [24, 25]. Nodal expression is significantly increased in human pancreatic cancer tissues and pancreatic cancer cell lines and is related to the high grade of pancreatic cancer. Knockdown Nodal expression reverses the invasive phenotype of pancreatic cancer and significantly decreases the number and size of liver metastases [18]. Ronaldo et al. examined pancreatic CSCs (cancer stem cells) from cell lines and primary tumor samples and found that they were highly enriched in Nodal/activin signals. Recombinant Nodal treatment enhances CSCs renewal and is blocked by the Alk receptor inhibitor SB431542 (specific to Alk4, Alk5, and Alk7) or the Nodal specific feedback inhibitor Lefty [26]. In our study, we found Nodal can affect the expression of MMP9 and promote the invasion and metastasis of pancreatic tumor cells. A previous study reported that Nodal plays a role in temporal and spatial neurodevelopment by regulating the mesoderm [27], but whether Nodal participates in pancreatic cancer PNI is unclear. So, we further studied the role of Nodal in the nerve invasion of pancreatic cancer.

Although PNI is an independent risk factor for pancreatic cancer, due to the complexity of the tumor microenvironment and insufficient understanding of PNI, there is almost no treatment for PNI. Previous studies showed the function of PNI may be affected by molecules (such as involving neurotrophies and their receptors, cytokines, chemokines, and neurotransmitters), metabolism (such as serine metabolism), and cellular mechanisms (such as involving Schwann cells and macrophages) [28–30]. The neurotrophic factor protein family includes NGF, BDNF, and GDNF, which can induce the survival, development, and function of neurons. They can also be produced and secreted by PDAC cells and directly affect the interaction between cancer cells and nerves in the tumor microenvironment through corresponding receptors. The interaction between tumor and nerve creates a microenvironment that is more suitable for tumor survival, thereby promoting tumor invasion and metastasis [31, 32]. For example, PDAC is exogenously dependent on serine. When serine is lacking, tumor cells can secrete NGF and act on nerve cells to increase the secretion of serine [33]. The combination of GDNF and GFRA1 (GDNF family receptor alpha-1) activates the RET signal. The GDNF-GFRA1-RET axis promotes cancer cell metastasis and matrix degradation by inducing cancer cell polarization and invasion pseudopodia [34]. The mechanism of tumor pain caused by pancreatic cancer is complicated. Tumor cell invasion destroys the normal structure of the nerve sheath and produces various molecules, leading to neuropathic and inflammatory pain. Neurotrophins can contribute to cancer pain directly. GDNF is related to the degree of pain in patients with pancreatic cancer [35]. By interacting with TRPV1 (transient receptor potential vanilloid 1), NGF can cause severe pain [36]. Our study finds that after rhNodal treatment, neurotrophins (NGF, BDNF, and GDNF) significantly increased in pancreatic cancer cells, and vice versa. The growth of DRGs treated with rhNodal was not significantly different from that in the control group. Next, we evaluated the function of Nodal in PNI progression using a DRG and pancreatic cancer cell coculture system. The nerve outgrowth ratio and tumor invasion index were higher in the rhNodal group compared with those of the control group. In contrast, knockdown of Nodal expression using siRNA reverses the interaction between DRGs and pancreatic cancer cells. These findings reveal that Nodal acts on tumor cells to promote the secretion of neurotrophins, thereby promoting the occurrence of nerve infiltration. Previous studies on neurodevelopment have shown that Nodal inhibits the differentiation of embryonic stem cells into the neuroectoderm directly and is indispensable in neurodevelopment and growth [27]. This finding may explain why the direct addition of rhNodal had no apparent effect on nerve growth, and the specific mechanism of its inhibitory function on nerve growth remains unclear.

Previous studies have shown that Nodal, expressed and secreted by pancreatic cancer stem cells and pancreatic stellate cells, plays an important role in maintaining the self-renewal and tumorigenicity of pancreatic cancer stem cells [33]. Our research has proved the role of Nodal in tumor invasion, metastasis, and neural invasion of pancreatic cancer, but the exact mechanism of Nodal affecting MMP9 and neurotrophic factors is still unclear. In addition, whether Nodal is a key step in exerting nerve infiltration and tumor metastasis, its role in tumor stem cells, pancreatic stellate cells, and nerve infiltration needs to be further explored.

## 5. Conclusions

Nodal is highly expressed in pancreatic cancer cells and promotes the invasive ability of tumor cells and enhances the trend of chemotactic infiltration to nerves during PNI. Activating Nodal signaling could increase neurotrophic factor expression in cancer cells and promote nerve growth and chemotaxis to cancer cells (Figure 5). New therapies that target Nodal may be useful in the treatment of PNI in pancreatic cancer.

## Figures and Tables

**Figure 1:** The effect of the Nodal signaling pathway on the interaction between pancreatic cancer cells and DRGs. (a) Compared with the control group, rhNodal promoted the trend of growth between DRGs and pancreatic cancer cells. (b) Compared with the NC group, siNodal by small interfering RNA significantly suppressed migration of Panc-1 and BxPC-3 cells toward DRG neurites. (c) The statistics and analysis of the invasion index and the DRG outgrowth index of the abovementioned grouping. (d) Illustration showing the calculation of the nerve invasion index (*α*/*γ*) and the DRG outgrowth ratio (*β*/*γ*). Magnification, ×100. ^*∗*/#^*P* < 0.05.

**Figure 2:** Nodal increases the expression of neurotrophins and enhances pancreatic cancer cell invasion. (a) Panc-1 and BxPC-3 cells were incubated with different concentrations of rhNodal (0, 50, and 100 *μ*M) for 24 h and western blot was used to evaluate NGF, BDNF, GDNF, and MMP-9 protein expression. (b) Panc-1 and BxPC-3 cells were pretreated with rhNodal (100 *μ*M) for 24 h and immunofluorescence analysis was conducted to assess the expression of NGF in Panc-1 and BxPC-3 cells. Magnification, ×400. (c) Panc-1 was treated with conditioned medium with different concentrations of rhNodal (0, 50, and 100 *μ*M) for 24 h; then, the supernatant of Panc-1 was collected and an ELISA was performed to evaluate the NGF level. (d) The effect of rhNodal on the invasive ability of Panc-1 and BxPC-3 cells was evaluated by the Matrigel invasion assay. Invasive cells were counted and plotted. Magnification, ×100. ^*∗*^*P* < 0.05.

**Figure 3:** Nodal knockdown decreases the expression of neurotrophins and inhibits pancreatic cancer cell invasion. (a) The efficiency of siRNAs targeting Nodal in PC cells was evaluated by western blotting assay. (b) Immunoblotting results revealed that knocking down Nodal expression restrained NGF, BDNF, GDNF, and MMP-9 protein expression. (c) NGF and Nodal are downregulated in both Panc-1 and BxPC-3 siNodal groups analyzed by immunofluorescence. Magnification, ×400. (d) The effect of the PC cell invasion capability was assessed using the Matrigel invasion assay. The invasion capability was significantly decreased in the group treated with siRNA compared with the NC group in Panc-1 and BxPC-3 cells. Magnification, ×100. ^*∗*^*P* < 0.05.

**Figure 4:** The growth of DRG synapses is Nodal-dependent. The outward growth of DRGs was observed under the microscope. After inhibition of Nodal by SB431542, compared with the rhNodal group, the invasive growth of DRGs was significantly reduced compared with the rhNodal group. Magnification, ×100. ^*∗*^*P* < 0.05.

**Figure 5:** Nodal is highly expressed in the pancreatic cancer microenvironment, promotes the invasion ability of tumor cells, and enhances the tendency of chemotactic infiltration to nerves in the process of PNI. Activating Nodal signaling could increase neurotrophic factor expression in cancer cells and promote nerve growth and chemotaxis to cancer cells.

## Data Availability

Data supporting the findings of this study are available from the corresponding authors upon reasonable request.

## Abbreviations

PNI: Perineural invasion
PDAC: Pancreatic ductal adenocarcinoma
NGF: Nerve growth factor
BDNF: Brain-derived neurotrophic factor
GDNF: Glial cell line-derived neurotrophic factor
TGF: Transforming growth factor
EMT: Epithelial-mesenchymal transition
MMPs: Matrix metalloproteinases
CSC: Cancer stem cell
DRG: Dorsal root ganglion
GFRA1: GDNF family receptor alpha-1
CTGF: Connective tissue growth factor
TRPV1: Transient receptor potential vanilloid 1.
